# Uterocervical angle versus cervical length in the prediction of spontaneous preterm birth in women with history of spontaneous preterm birth: a prospective observational study

This article has been retracted.

**DOI:** 10.1186/s12884-023-05977-9

**Published:** 2023-09-13

**Authors:** Ahmed Mohammed Elmaraghy, Salma Mohamed Ahmed Shaaban, Mohammed Salah Elsokkary, Ibrahim Shazly Mohamed Amen Elshazly

**Affiliations:** 1 Department of Obstetrics and Gynecology, Faculty of Medicine, Ain Shams University, Cairo, Egypt; 2 Alexandria specialized hospital, Ministry of health, Alexandria, Egypt

**Keywords:** Preterm birth, Anterior uterocervical angle, Cervical length

## Abstract

**Background:**

Preterm delivery is a leading cause of neonatal mortality and morbidity. History of spontaneous preterm birth is the greatest risk factor for another preterm delivery. So, every effort should be made to prevent the recurrence of preterm delivery in this vulnerable group. This study aimed to evaluate the predictive ability of the anterior uterocervical angle and cervical length in preterm birth.

**Patients and Methods:**

This was a prospective cohort study that included 70 patients with a history of spontaneous preterm birth. Ultrasound measurements of cervical length and anterior uterocervical angle were set to be measured for each patient at three visits; first between 16 ^0/7^ and 24 ^0/7^ weeks, second between 24 ^1/7^ and 32 ^0/7^ weeks, and the third was between 32 ^1/7^ and 36 ^6/7^ weeks. The correlation between both measures and the prediction of preterm birth among study participants was the primary outcome of the study. Neonatal outcome among the study patients was a secondary measure of outcome.

**Results:**

The incidence of preterm birth among study participants was 31.41%. Cervical length and uterocervical angle showed progressive decrease and increase respectively throughout pregnancy. At the 2^nd^ visit, the two measures were significantly different between those who delivered at term and those with preterm delivery with the cervical length being significantly shorter in the preterm arm (3.0 ± 0.49 versus 3.38 ± 0.36, *p* < 0.001) and uterocervical angle being significantly bigger among the same arm (110.1 ± 18.48 versus 84.42 ± 12.24, *p* < 0.001). A uterocervical angle > 89.8° at the second visit predicted preterm birth with 81.8% sensitivity and 70.8% specificity while cervical length ≤ 3.22 cm at the second visit predicted preterm birth with 68.1% sensitivity and 62.5% specificity. Multivariant logistic regression analysis showed that uterocervical angle > 89.8° at the second visit increased the odds ratio for preterm birth by 9.

**Conclusion:**

Uterocervical angle can be a useful ultrasound marker for the prediction of preterm birth among high risk patients. A cutoff value of 89.8° can be used as a threshold above which prophylactic measures such as cervical cerclage or progesterone therapy can be provided.

**Trial registration:**

NCT05632003 (First posted date: 30/11/2022).

## Introduction

Preterm birth (PTB) is a major cause of neonatal morbidity and mortality. Annually, nearly one million babies die due to adverse events caused by prematurity [1]. Preterm birth is defined by the WHO as all births before 37 completed weeks of gestation, or fewer than 259 days from the first date of a woman’s last menstrual period [2]. Preterm delivery is further divided into three categories; very early preterm (before 32 weeks), early preterm (32 ^0/7^ to 33 ^6/7^ weeks), and late preterm (34 ^0/7^ to 36 ^6/7^ weeks) [3].

The etiology behind preterm birth is poorly understood. It’s believed to be multi-factorial with obstetric, environmental, demographic, and genetic factors likely to be involved in the pathophysiology either separately or synergistically [4]. Along the many risk factors that are associated with preterm delivery, previous history of spontaneous preterm birth remains the leading and most recognized one and so, a such critical group needs to be properly identified to provide proper pre-conceptional and antenatal care for subsequent pregnancies [5].

Preterm infants are at increased risk of a wide range of complications as respiratory distress syndrome, necrotizing enterocolitis, and neonatal sepsis. Long term morbidities such as sensory and motor deficits, cognitive impairment, and behavioral complications are more common in babies who were born preterm compared with those who were born at term [6]. Consequently, effective prophylactic measures are needed to minimize the morbidities and complications associated with preterm birth as much as possible. Developing effective prevention of preterm labor can be achieved by throughout knowledge of the epidemiology of preterm birth and the risk factors associated with it [7].

Preventive measures can be offered to patients who are at high risk of preterm labor and so, screening for these patients in asymptomatic women is crucial [8]. Many prophylactic strategies have been suggested; universal screening by cervical length for all pregnant followed by progesterone therapy or cerclage has been implemented by many institutes, and smoking cessation programs can be of great value as well [9].

Cervical length assessment in the second trimester through transvaginal ultrasound assessment is a strong predictor for spontaneous preterm birth. Cervical length ≤ 25 mm at 22 + 0 to 24 + 6 weeks of gestation has been associated with 37.3% sensitivity, 92.2% specificity, 17.8% positive predictive value, and 97.0% negative predictive value for the prediction of spontaneous preterm birth at < 35 weeks of gestation [10]. The Anterior uterocervical angle is defined as the angle between the cervix and the anterior uterine wall; this angle can be measured by ultrasound and its width can be of great value in predicting preterm birth. The importance of this angle in the prediction of preterm birth comes from the fact that any force applied to the uterus while the angle is acute will increase the closure force of the cervix whereas an obtuse angle will eventually open the cervix. It has been suggested that using both cervical length and anterior uterocervical can predict preterm birth with great accuracy [11].

Our study aims to compare between sonographic measurements; the cervical length and the uterocervical angle regarding their ability to predict spontaneous preterm birth.

### Patients & Methods

This prospective observational study was conducted at Ain Shams University Maternity Hospital during the period from January 2022 to December 2022. Before the initiation of the study, approval of the Ethical Committee of the Faculty of Medicine, Ain Shams University was obtained (MS 634/2021, FWA 000017585). Using the PASS II program for sample size calculation; setting power at 90% and α – error at 0.05 and according to previous literature, the expected sensitivity of Uterocervical angle and Cervical length for prediction of preterm birth was 86% and 28% respectively with 27% incidence of preterm birth [11]; a minimum sample size of 70 patients was needed to detect the difference in the predictive ability between the two measures. The study participants were seventy pregnant women with singleton pregnancy and history of spontaneous preterm birth. The study was registered at ClinicalTrials.gov (ID: NCT05632003), (First posted date: 30/11/2022).

Age of the included participants ranged from 18 to 35 years. Normal fetal growth pattern by fetal biometry and estimated fetal weight was a prerequisite for inclusion in the study. Patients with risk factors for preterm delivery apart from the past history of spontaneous preterm birth as medical disorders associated with uteroplacental insufficiency, congenital uterine anomalies, congenital fetal malformations, preterm pre-labor rupture of membranes, polyhydramnios, and those with threatened abortion or antepartum hemorrhage during the present pregnancy were excluded from the study. Moreover, patients who had cervical cerclage during the present pregnancy and those with history of cervical trauma (cervical conization) were also excluded from the study.

Informed consent was taken from study participants before enrollment and after a thorough explanation of the purpose of the study. All patients included in the study were recruited at 16 – 24 weeks of gestation when history taking, physical examination, and detailed anomaly scan were done to ensure that each patient met our inclusion / exclusion criteria. Cervical length and uterocervical angle were set to be measured on three occasions; the first between 16 ^0/7^ to 24 ^0/7^ weeks of gestation, the second between 24 ^1/7^ and 32 ^0/7^ weeks of gestation, and the third between 32 ^1/7^ and 36 ^6/7^ weeks of gestation. For each patient, a minimum of 4 weeks between each visit was ensured. As our patients were recruited from 16 – 24 weeks of gestation, not all of them had early scans to depend on it for gestational age calculation. We depended on the date of last menstrual period for calculation of gestational age and estimated gestational age obtained from the ultrasound performed at the first visit corresponded to menstrual dating.

The cervical length was measured as follows; a sagittal view of the cervix was required, the cervical canal with the surrounding mucosa was identified, the isthmus wasn’t included, visualization of both external and internal os was ensured, the image was magnified to a degree that the cervix occupied 50–75% of it, and measurement was taken by placing the calipers between the external and the internal os [12]. As for the anterior uterocervical angle, the vaginal probe was inserted till reaching the anterior fornix. A longitudinal view of the cervix was obtained for the entire length of the cervical canal to be visualized. Then, the image was magnified so that the cervix can occupy about two thirds of the screen. The anterior uterocervical angle is defined as the angle measured between the lower uterine segment and the cervical canal. A straight line was traced between the external os and the internal os, including the isthmus. Another line, 3 cm long, was traced parallel to the lowest part of the anterior uterine wall. The angle created by the intersection of the two lines (aUCA) was measured [13]. Ultrasound assessment was performed by an Obstetrics and Gynecology (OB/GYN) consultant with special interest in fetal medicine and OB/GYN ultrasound. All scans were performed at the Ultrasound and Fetal Care Unit, Ain Shams University Maternity hospital. Both CL and aUCA were measured simultaneously and plotted on a chart to identify a cutoff value with accepted sensitivity and specificity for predicting preterm birth; Cervical length ≤ 25 mm was the cutoff values for initiation of progesterone therapy. Figures 1, 2 and 3 represent three measurements of the uterocervical angle for the same patient obtained at the three consecutive visits; this patient was 30 years old, G4, P2 CS + 1 and her last pregnancy was complicated by spontaneous preterm delivery at 35 weeks which led to emergency CS yielding living male which was admitted to the NICU for 6 days then discharged. As shown in the figures, there was progressive increase in the uterocervical angle and eventually the patient underwent late preterm birth at 36 wks.

**Fig.1:** Uterocervical angle at the first visit (23wks + 4 days): 97.6°

**Fig.2:** Uterocervical angle at the second visit (28wks): 118.96°

**Fig.3:** Uterocervical angle at the third visit (32wks + 1day): 128.65°

The correlation between both measures and prediction of preterm birth before completed 37 weeks of gestation among study participants was the main target of the study. Neonatal outcome among the study patients was a secondary measure of outcome.

Regarding the statistical analysis, quantitative variables were presented using mean and standard deviation, qualitative variables were presented using count and percentage. Student t-test was used to compare quantitative variables between two independent groups, Chi square test was used for qualitative variables, Mann Whitney test was used to compare the two arms of the study for abnormally distributed quantitative variables, Fisher’s Exact or Monte Carlo correction was used for correction for chi-square when more than 20% of the cells have expected count less than 5, ROC curve analysis was used to compare the predictive ability of the two measures and determine the best cut off value with the highest sensitivity and specificity for each measure, Logistic regression analysis was done to measure the ability of different factors for prediction of preterm birth, and P value less than or equal to 0.05 was considered statistically significant.

## Results

The study was conducted at Ain Shams University Maternity Hospital. 77 patients were enrolled in the study; 7 patients were excluded after enrollment with 4 patients refused to adhere to the study protocol, 2 patients developed membrane rupture and one patient had threatened abortion. Seventy patients attended both 1^st^ and 2^nd^ visits while only 52 patients attended the 3^rd^ visit; the 18 patients who didn’t attend the third visit delivered preterm with 5 patients had a very early preterm delivery before the start of the visit, and 13 patients delivered either early preterm or late preterm ie after the start of the visit **(**Fig. 4**).**

**Fig. 4:** Flow chart of pathway of enrolled participants

Among the study participants, the incidence of preterm birth was 31.4%; out of the 22 cases who delivered preterm, 5 cases had a very early preterm birth (before 32 weeks), 7 cases had an early preterm birth (32 ^0/7^ to 33 ^6/7^ weeks), and 10 cases had late preterm birth (34 ^0/7^ to 36 ^6/7^ weeks) **(**Table 1**).**

**Table 1:** Distribution of cases according to the incidence of preterm birth (*n* = 70)

Incidence of preterm birth		%
22/70		**31.4%**
Very early	**5**	**7.1%**
Early	**7**	**10%**
Late	**10**	**14.3%**

The demographic data of the study participants was presented in Table 2. All the study participants had a history of ≥ 1 spontaneous preterm birth. Seventy participants attended both the 1^st^ and 2^nd^ visits while 52 patients attended the third visit because the remaining 18 patients either delivered prior to the visit or didn’t attend. At each visit, cervical length and uterocervical angle were measured. Table 3 showed that there was a progressive decline in cervical length with advancing gestational age while Table 4 showed progressive increase in uterocervical angle with advance in gestational age. The mode of delivery among the study patients was shown in Table 5.

**Table 2:** Demographic data of the studied population

	**Total (*n *= 70)**		**Incidence of preterm birth**				**Test of significance**	***P***
			**Yes (*n* = 22)**		**No (*n* = 48)**			
**Age (years)**								
**Mean ± SD**	**26.03 ± 4.43**		**26.27 ± 4.81**		**25.92 ± 4.29**		**t = 0.310**	**0.757 (NS)**
**BMI (Kg/m2)**								
**Mean ± SD**	**27.38 ± 3.52**		**27.40 ± 3.43**		**27.37 ± 3.60**		**t = 0.032**	**0.975 (NS)**
**Parity**								
**Min – Max**	**1.0 – 5.0**		**1.0 – 5.0**		**1.0 – 4.0**		**U = 502.0**	**0.724 (NS)**
**Median (IQR)**	**2.0 (1.0 – 2.0)**		**2.0 (1.0 – 2.0)**		**2.0 (1.0 – 2.0)**			
**Past CS**	**No**	**%**	**No**	**%**	**No**	**%**		
**No**	**45**	**64.3**	**13**	**59.1**	**32**	**66.7**	**χ**^**2**^** = 0.377**	**0.539 (NS)**
**Yes**	**25**	**35.7**	**9**	**40.9**	**16**	**33.3**		
**Pre-delivery Hemoglobin**								
**Mean ± SD**	**11.27 ± 0.92**		**11.34 ± 0.85**		**11.24 ± 0.96**		**t = 0.398**	**0.692 (NS)**

*SD* Standard deviation, *IQR* Interquartile range, *t* Student t-test, *U* Mann Whitney test, χ^2^ Chi square test, *NS* Non-significant, *p* p value

**Table 3:** Cervical length among the study participants

Cervical length (cm)	Total (*n* = 70)	Incidence of preterm birth		Test of significance	*P*
		**Yes (*n *= 22)**	**No (*n* = 48)**		
**1**^**st**^** visit**					
**Mean ± SD**	**3.75 ± 0.51**	**3.60 ± 0.60**	**3.81 ± 0.45**	**t = 1.681**	**0.097 (NS)**
**2**^**nd**^** visit**					
**Mean ± SD**	**3.26 ± 0.44**	**3.0 ± 0.49**	**3.38 ± 0.36**	t = 3.715^*^	< 0.001* (S)
**3**^**rd**^** visit**	**(n = 52)**	**(n = 4)**	**(n = 48)**		
**Mean ± SD**	**3.01 ± 0.33**	**2.94 ± 0.42**	**3.02 ± 0.33**	**t = 0.452**	**0.653 (NS)**

*SD* Standard deviation, *t* Student t-test, *p* p value, *: statistically significant at *p* ≤ 0.05

1^st^ visit: 16 ^0/7^ weeks – 24 ^0/7^ weeks

2^nd^ visit: 24 ^1/7^ weeks – 32 ^0/7^ weeks

3^rd^ visit: 32 ^1/7^ weeks – 36 ^6/7^ weeks

**Table 4:** Uterocervical angle among the study participants:

Uterocervical angle ( °)	Total (*n* = 70)	Incidence of preterm birth		Test of significance	*P*
		**Yes (*n* = 22)**	**No (*n* = 48)**		
**1**^**st**^** visit**					
**Mean ± SD**	**81.51 ± 17.10**	**93.32 ± 19.09**	**76.10 ± 13.09**	**t = 3.839**	0.001* **(S)**
**2**^**nd**^** visit**					
**Mean ± SD**	**92.48 ± 18.71**	**110.1 ± 18.48**	**84.42 ± 12.24**	**t = 5.943**	< 0.001* **(S)**
**3**^**rd**^** visit**	**(*n* = 52)**	**(*n* = 4)**	**(*n* = 48)**		
**Mean ± SD**	**96.39 ± 14.75**	**123.3 ± 23.16**	**94.15 ± 11.63**	**t = 2.489**	**0.085 (NS)**

*SD* Standard deviation, *t* Student t-test, *p* p value, *: statistically significant at *p* ≤ 0.05

1^st^ visit: 16 ^0/7^ weeks – 24 ^0/7^ weeks

2^nd^ visit: 24 ^1/7^ weeks – 32 ^0/7^ weeks

3^rd^ visit: 32 ^1/7^ weeks – 36 ^6/7^ weeks

**Table 5:** Mode of delivery among the study participants

Mode of delivery	Total (*n* = 70)		Incidence of preterm birth				Test of significance χ^2^	^MC^P
	**No**	**%**	**Yes (*n* = 22)**		**No (*n* = 48)**			
			**No**	**%**	**No**	**%**		
**Cesarean section**	**36**	**51.4%**	**10**	**45.5%**	**26**	**54.2%**	**0.701**	0.822 (NS**)**
**Vaginal delivery**	**31**	**44.3%**	**11**	**50%**	**20**	**41.7%**		
**VBAC**	**3**	**4.3%**	**1**	**4.5%**	**2**	**4.1%**		

**χ**^**2**^ Chi-square test, ***MC*** Monte carlo, *p* p value

Table 6 compared both arms of the study regarding gestational age when delivery occurred; there was a significant difference between the two arms favoring the term arm. Table 7 showed the neonatal outcome among the study participants; 45 neonates were discharged within the first 24 h after delivery (41 neonates from the term arm and 4 neonates from the preterm arm), 7 neonates from the preterm arm died at the NICU while 18 neonates were discharged after NICU admission (11 from the preterm arm and 7 from the term arm).

**Table 6:** Gestational age at delivery among the study participants

Gestational age at delivery (weeks)	Total (*n* = 70)	Incidence of preterm birth		t	p
		**Yes (*n* = 22)**	**No (*n* = 48)**		
**Mean ± SD**	**37.00 ± 2.62**	**33.84 ± 2.21**	**38.45 ± 0.84**	**9.483**	< 0.001^*^

*SD* Standard deviation, *t* Student t-test, *p* p value for comparing between term and preterm

^*^Statistically significant at *p* ≤ 0.05

**Table 7:** Neonatal outcome of the study participants

**Neonatal outcome**	**Total (*n* = 70)**		**Incidence of preterm birth**				**Test of significance** **χ**^**2**^	^**MC**^**P**
	**No**	**%**	**Yes (*n* = 22)**		**No (*n* = 48)**			
			**No**	**%**	**No**	**%**		
**Discharged within the first 24 h**	**45**	**64.3%**	**4**	**18.2%**	**41**	**85.4%**	**33.028**	< 0.001* **(S)**
**NICU admission (Died)**	**7**	**10%**	**7**	**31.8%**	**0**	**0.0%**		
**NICU admission (Discharged)**	**18**	**25.7%**	**11**	**50%**	**7**	**14.6%**		

**χ**^**2**^ Chi-square test, *MC* Monte carlo, *p* p value, *statistically significant at *p* ≤ 0.05

The accuracy of cervical length and uterocervical angle in predicting preterm birth was assessed at the 3 visits; Fig. 5 represented the ROC curve of both measures at the 1^st^ visit while Fig. 6 represented the ROC curve at the 2^nd^ visit while a ROC curve for the third visit was not possible since only 4 patients from the preterm arm attended the third visit i.e. the start of the third visit. Table 8 showed that cervical length ≤ 3.67 mm during the period from 16 ^0/7^ to 24 ^0/7^ weeks of gestation was associated with 63.64% sensitivity, 62.50% specificity, 43.7% PPV, and 78.9% NPV, while uterocervical angle > 81° during the same gestational age was associated with 72.73% sensitivity, 64.58% specificity, 48.5 PPV %, and 83.8% NPV. Table 9 showed that cervical length ≤ 3.22 mm during the period from 24 ^1/7^ and 32 ^0/7^ weeks of gestation was associated with 68.18% sensitivity, 62.50% specificity, 45.5% PPV, and 81.1% NPV, while uterocervical angle > 89.81° during the same gestational age was associated with 81.82% sensitivity, 70.83% specificity, 56.3% PPV, and 89.5% NPV. Table 10 showed that among the study participants, cervical length and uterocervical angle during the gestational age of 2^nd^ visit were independent risk factors for spontaneous preterm birth, however, the only significant variable was anterior uterocervical angle > 89.9° with an odds ratio of 9 for spontaneous preterm birth.

**Fig. 5:** ROC curve for Cervical length and Uterocervical angle to predict preterm birth at 1.^st^visit (*n* = 22 vs. 48)

**Fig. 6:** ROC curve for Cervical length and Uterocervical angle to predict preterm birth at 2.^nd^ visit (*n* = 22 vs. 48)

**Table 8:** Validity (AUC, sensitivity, specificity) for cervical length and uterocervical angle to predict preterm birth at 1^st^visit (*n* = 22 vs. 48)

At 1^st^ Visit	AUC	P	95% CI	Cut off	Sensitivity	Specificity	PPV	NPV
Cervical length (mm)	**0.619**	**0.112**	**0.465—0.773**	** ≤ 3.67**	**63.64**	**62.50**	**43.7**	**78.9**
Cervical length (mm)				< 2.45**	**0.00**	**100.00**		**68.6**
Cervical length (mm)				≤ 2.79**	**9.09**	**100.00**	**100.0**	**70.6**
Uterocervical Angle ( °)	**0.752**	0.001*	**0.616– 0.888**	** > 81**	**72.73**	**64.58**	**48.5**	**83.8**

*AUC* Area under curve, *CI* Confidence intervals, *PPV* positive predictive value, *NPV* Negative predictive value, *statistically significant at *p* ≤ 0.05

^**^These cutoff values are added for comparison as the nearest values in the study population to the standard 25-mm cutoff for short cervix

**Table 9:** Validity (AUC, sensitivity, specificity) for cervical length and uterocervical angle to predict preterm birth at 2^nd^ visit (*n = *22 vs. 48)

At 2^nd^ Visit	AUC	P	95% CI	Cut off	Sensitivity	Specificity	PPV	NPV
Cervical length (mm)	**0.743**	0.001*	**0.609—0.877**	** ≤ 3.22**	**68.18**	**62.50**	**45.5**	**81.1**
Cervical length (mm)				≤ 2.56**	**13.64**	**100.00**	**100.00**	**71.6**
Uterocervical Angle ( °)	**0.866**	< 0.001*	**0.761 – 0.971**	** > 89.81**	**81.82**	**70.83**	**56.3**	**89.5**

*AUC* Area under curve, *CI* Confidence intervals, *PPV* Positive predictive value, *NPV* Negative predictive value, *: statistically significant at *p* ≤ 0.05

^**^This cutoff value is added for comparison as the nearest value in the study population to the standard 25-mm cutoff for short cervix

**Table 10:** Univariate and multivariate logistic regression analysis for the parameters affecting incidence of preterm birth (*n* = 22 vs. 48)

	**Univariate**		^**#**^**Multivariate**	
	***p***	**OR (LL – UL 95%C.I)**	***p***	**OR (LL – UL 95%C.I)**
**Age (years)**	0.753	1.019 (0.908 – 1.143)		
**BMI (kg/m**^**2**^**)**	0.974	1.002 (0.868 – 1.158)		
**Hemoglobin**	0.687	1.120 (0.645 – 1.945)		
**Parity**	0.360	1.265 (0.765 – 2.090)		
**Cervical length 1**^**st**^** visit**	0.089	0.393 (0.134 – 1.155)		
**Cervical length 2**^**nd**^** visit (≤ 3.22)**	0.020^*^	3.571 (1.224 – 10.419)	0.155	2.425 (0.716 – 8.216)
**Anterior uterocervical angle 1**^**st**^** visit (> 81)**	0.005^*^	4.863 (1.604 – 14.743)	0.984	1.019 (0.169 – 6.155)
**Anterior uterocervical angle 2**^**nd**^** visit (> 89.81)**	< 0.001^*^	10.929 (3.133 – 38.124)	0.020^*^	9.093 (1.421 – 58.19)

*OR* Odd`s ratio, *C.I* Confidence interval, *LL* Lower limit, *UL* Upper Limit

^*^Statistically significant at *p* ≤ 0.05

Regarding progesterone therapy, cervical length < 25 mm was reported in 8 patients who were instructed to receive vaginal progesterone immediately after the test; 3 out of 8 patients delivered preterm while the remaining 5 patients delivered at term.

## Discussion

This prospective study was conducted during the period from January 2022 to December 2022. Seventy patients with a past history of spontaneous preterm birth met the inclusion / exclusion criteria and three visits were scheduled for each one of the study participants during which, the cervical length and the anterior uterocervical angle were measured. The outcome of the study divided the study participants into two arms; the first arm represented the participants who delivered at term while the second arm represented those who eventually had spontaneous preterm delivery.

Regarding the demographic data, there was no significant difference between the two arms regarding age, parity, BMI, history of previous cesarean section, and pre-delivery hemoglobin. The mean hemoglobin level in both groups was ≥ 10 g/dl which reflected that maternal anemia was not a hidden risk factor for preterm birth in our study.

The incidence of preterm birth in our study was 31.4%. A such relatively high percentage was attributed to the nature of the study participants as they all had a past history of at least one spontaneous preterm birth which is the greatest risk factor for preterm birth.

The cervical length decreased with the advance in gestational age; this finding was observed in those who delivered at term and those who had preterm delivery. Cervical length was shorter among those who delivered preterm compared to the term arm at visits 1 and 2 with statistical significance being observed only at the second visit i.e. from 24 ^1/7^ weeks – 32 ^0/7^ weeks of gestation. Our results were similar to those obtained by Abuelghar et al., who showed in their cohort study that cervical length decreased as pregnancy progressed among the three arms of their study; those who delivered at term, late preterm, and early preterm; the study participants underwent assessment of cervical length on two occasions 3–4 weeks apart with the first assessment being carried out at 24–28 weeks of gestation [14]. The results were also similar to those obtained by Esplin et al., who conducted their study on nulliparous women aiming for identifying the predictive accuracy of both cervical length and fetal fibronectin; the study participants offered 3 visits at least 4 weeks apart when the cervical length was measured at visits 2 and 3. Transvaginal cervical length decreased to a greater degree between visits 2 and 3 among those who delivered preterm [15].

Regarding anterior uterocervical angle, it became wider with the progression of gestational age in both arms of the study and it was bigger among those who delivered preterm during the three visits with statistical significance observed at 1^st^ and 2^nd^ visits. Our results were similar to those obtained by Sawaddisan et al., who assessed uterocervical angle on patients with normal cervical length and no history of preterm birth during gestational age from 16 ^0/7^ weeks to 24 ^0/7^ weeks; a wider uterocervical angle was observed among those who delivered preterm but with statistical significance in those who were assessed at 19.5 – 24 ^0/7^ weeks [16]. The results obtained by Gründler et al., were inconsistent with our results as there was no difference in uterocervical angle measured during the period from 20 ^0/7^ weeks to 31 _6/7_ weeks between those who delivered after 37 weeks and those with preterm delivery; such inconsistency in results can be attributed to the nature of the study participants as the authors included patients with threatened preterm labor, cervical length less than 25 mm, and multiple gestations; such factors could affect the uterocervical angle making it wider even in those who delivered at term [17].

There was no significant difference between both arms of the study regarding the mode of delivery with 54.2% of cases from the term arm delivered by cesarean section while the cesarean section was present at 45.5% of cases from the preterm arm. Such a high rate of cesarean section in our study can be attributed to two factors; history of a previous cesarean section which was present in 40.9% of patients from the preterm arm and 33.3% of patients from the term arm, and the fact that our hospital is considered a high volume tertiary OB/GYN center but with limited resources such as electronic fetal monitoring devices which limits continuous fetal monitoring during labor for high risk patients. Our results were similar to those obtained by Sawaddisan et al., who had a 57.4% cesarean rate in the term arm and a 44.1% cesarean rate in the preterm arm [16]. The study was conducted at a tertiary hospital in southern Thailand, and almost 25% of the participants from the term arm and 35% of the preterm arm had a history of previous cesarean section; such factors could explain the high rate of cesarean section in this study.

Gestational age when delivery occurred was evaluated and it was significantly higher among the term arm; Singh et al., had a higher mean gestational age at delivery for the preterm group compared to our study (35.5 vs 33.8); this can be attributed to the nature of the study participants being low risk patients with no risk factors for preterm delivery [18]. Gründler et al., obtained slightly lower mean gestational age at delivery for the preterm group compared to our study (32.1 vs 33.8); this can be explained by the presence of patients with threatened preterm labor, short cervical length (< 25 mm), and multiple pregnancy among the included participants [17].

The neonatal outcomes among the study participants were assessed; there was a significant difference between the two arms of the study with 85.4% of the neonates from the term arm being discharged within 24 h versus 18.2% of the neonates from the preterm arm. Neonatal mortality was present in 31.8% of the neonates from the preterm arm while none of the term neonates suffered neonatal mortality; Four out of these seven neonatal mortalities were due to respiratory distress syndrome while the remaining three suffered from neonatal sepsis. Algameel et al., assessed the outcome of late preterm newborns in Upper Egypt; 52.9% of the late preterm newborns were admitted to the neonatal intensive care unit [19]. Such a percentage is lower compared to our study as the study was limited to late preterm newborns. Half of the preterm neonates of our study were discharged after a period of NICU admission; they were admitted for different reasons including neonatal jaundice (45.4%), respiratory distress syndrome (27.3%), neonatal hypoglycemia (18.2%), and birth asphyxia (9.1%).

The predictive accuracy of both cervical length and uterocervical angle for preterm birth was assessed; the ROC curve showed a bigger area under the curve (AUC) for the uterocervical angle at both 1^st^ and 2^nd^ visits. During the second visit, the predictive accuracy for both measures increased; however, the uterocervical angle retained higher sensitivity, specificity, PPV, and NPV **(**Table 9**)** The multivariant logistic regression analysis showed that during the 2nd visit, cervical length less than 3.22 mm was associated with an odds ratio of 2.4 for spontaneous preterm birth while anterior uterocervical angle > 89.8 was associated with an odds ratio of 9 for spontaneous preterm birth among study participants. The overlapping CI for AUC indicate that the AUCA may not be consistently outperforming CL, however AUCA might provide better prediction according to the point estimate. This may be elucidated with further studies with larger sample size. Our results were similar to those obtained by Khamees et al., who assessed the diagnostic performance of both cervical length and uterocervical angle at three visits; 30 – 32, 32 ^+1^ – 34, and 34^+1^ – 36 ^+1^ weeks, the diagnostic performance of uterocervical angle was similar to our results at the second visit but with higher cutoff value (105° vs 89.9°) [11]. This higher cutoff value can be attributed to the gestational age when the measures were obtained which was more advanced than our study, and the fact the study participants were a heterogeneous cohort including patients with any risk factor for preterm birth in contrast to our study which targeted patients with history of spontaneous preterm birth which is the greatest risk factor for spontaneous preterm delivery. Regarding the cervical length, the lower sensitivity and higher specificity compared to our study can be attributed to the higher cutoff value in our study (3.22 cm vs 2.5 cm). Dziadosz et al., assessed the diagnostic performance of the uterocervical angle measured during the period from 16 ^0/7^ to 23 ^6/7^ weeks for prediction of spontaneous preterm birth; compared with the results obtained from our 1^st^ visit, a similar AUC was obtained (0.78 vs 0.75) but a higher cutoff value for prediction of spontaneous preterm birth (95° vs 81°), however, higher sensitivity and lower specificity compared to our study were reported which can be attributed to much higher sample size and lower incidence of spontaneous preterm birth among study participants (972 vs 70) and ( 9.6% vs 31.4%) respectively [20]. The two previously mentioned studies were in line with our study in concluding that uterocervical angle is more predictive of spontaneous preterm birth compared with cervical length [11, 20]. Luechathananon et al., assessed the predictive accuracy of both measures in patients with threatened preterm labor; a cervical length < 3.4 cm was associated with 72.1% sensitivity, 46.2% specificity, 33% PPV, and 81.1% NPV for predicting preterm birth [21]. The higher sensitivity compared to our results obtained from the measures of our 1st visit can be attributed to the gestational age when the measures were taken being higher than our study (median gestational age was 33 weeks) while the sensitivity was very close when measures were compared with the second visit (72.1% vs 68.1%). Regarding the uterocervical angle, an acute angle reinforces the closure of the endocervical canal, while a more obtuse angle may facilitate the opening of the cervix [22]; this could be the reason why Luechathananon et al., obtained a higher cutoff value compared to our study (110.97° vs 89.81° or 81) [21]. In contrast to our study, results obtained by Wagner et al., showed that the uterocervical angle is not a useful measure for the prediction of preterm birth, the included patients in this study accounted for that difference as they included patients with regular uterine contractions and cervical length less than 25 mm which indicated a very high risk for preterm delivery; an obtuse uterocervical angle was predominant in the three study groups that were delivery within 2 days, 3–7 days and after 7 days with corresponding median UCA angle of 108.5, 108°, and 107.3° [23]. The value of these findings is that when it comes to patients with already established uterine contractions and cervical changes, the value of the uterocervical angle in predicting preterm delivery is questioned. Sawaddisan et al., showed that the uterocervical angle is not a good predictor of spontaneous birth; however, the study participants were at low risk for spontaneous preterm birth with no history of neither spontaneous preterm birth nor second trimesteric miscarriage [16]. The value of the anterior uterocervical angle among patients with low risk for spontaneous preterm birth needs further future studies with large sample size for better identification of its value.

Regarding progesterone therapy, only 8 patients (11.4%) from the study cohort had cervical length less than 25 mm during the follow up visits and consequently received progesterone therapy; a higher sample size is needed for better evaluation of the effect of progesterone in patients with short cervix.

Our study was not without limitations; we weren’t able to determine a cutoff value for those who attended the third visit due to the fact that only 4 patients from those who attended the third visit (*n* = 52) delivered preterm; a bigger sample size will be needed in future studies to determine a cutoff value for the uterocervical angle for patients who are between 32 and 37 weeks.

Uterocervical angle appears to be a good predictor for spontaneous preterm birth among patients with history of spontaneous preterm birth. Combination of both cervical length and anterior uterocervical angle as screening tests for preterm birth among high risk patients may provide better predictive accuracy than cervical length alone.

## Conclusion

Anterior uterocervical angle is a useful ultrasound marker which can be incorporated in the screening workup of pregnant women with history of previous spontaneous preterm birth. A cutoff of 89.8° can be used in future studies to evaluate whether prophylactic treatment for women with past history of preterm birth will be effective in reducing the incidence of preterm birth in such high risk cohort.

## Data Availability

The datasets used and/or analyzed during the current study are available from the corresponding author on reasonable request.
